# Simulation Analysis of the Aerodynamic Performance of a Bionic Aircraft with Foldable Beetle Wings in Gliding Flight

**DOI:** 10.1155/2020/8843360

**Published:** 2020-12-24

**Authors:** Caidong Wang, Yu Ning, Xinjie Wang, Junqiu Zhang, Liangwen Wang

**Affiliations:** ^1^College of Mechanical and Electrical Engineering, Zhengzhou University of Light Industry, Zhengzhou 450002, China; ^2^Henan Key Laboratory of Intelligent Manufacturing of Mechanical Equipment, Zhengzhou 450002, China; ^3^Key Laboratory of Bionic Engineering, Ministry of Education, Jilin University, Changchun 130022, China

## Abstract

Beetles have excellent flight performance. Based on the four-plate mechanism theory, a novel bionic flapping aircraft with foldable beetle wings was designed. It can perform flapping, gliding, wing folding, and abduction/adduction movements with a self-locking function. In order to study the flight characteristics of beetles and improve their gliding performance, this paper used a two-way Fluid-Structure Interaction (FSI) numerical simulation method to focus on the gliding performance of the bionic flapping aircraft. The effects of elastic model, rigid and flexible wing, angle of attack, and velocity on the aerodynamic characteristics of the aircraft in gliding flight are analyzed. It was found that the elastic modulus of the flexible hinges has little effect on the aerodynamic performance of the aircraft. Both the rigid and the flexible wings have a maximum lift-to-drag ratio when the attack angle is 10°. The lift increased with the increase of the gliding speed, and it was found that the lift cannot support the gliding movement at low speeds. In order to achieve gliding, considering the weight and flight performance, the weight of the microair vehicle is controlled at about 3 g, and the gliding speed is guaranteed to be greater than 6.5 m/s. The results of this study are of great significance for the design of bionic flapping aircrafts.

## 1. Introduction

Most insects and birds in nature have excellent flight performance [1, 2]. In the evolutionary history of life on Earth, insects were the first to acquire flying skills, at least 50 million years earlier than reptiles and birds. Although many insects are small in size, they exhibit superb flying skills and flexible maneuverability. After more than 20 years of development, various MAVs (Micro Air Vehicles) with different functions have been designed and developed. Depending on the flight mode, MAVs can be divided into fixed-wing aircrafts, rotor-wing aircrafts, and flapping-wing aircrafts [3]. The flight principle and design of the fixed-wing and rotor-wing MAVs are similar to those of conventional aircrafts. Thanks to the technological evolution of conventional aircrafts, the fixed-wing and rotor-wing MAVs have become the main direction of MAV research. However, the development of flapping-wing aircrafts has benefited from the interactive integration of bionics and multidisciplinary interaction. They are of the same order of magnitude, with a comparable Reynolds number, and fully in line with the prototype requirements of MAV design. Flapping-wing MAVs have been developed to mimic the flight patterns of birds and insects. However, the development of flapping-wing aircrafts has benefited from the interactive integration of bionics and multidisciplinary interaction. Flapping-wing MAVs have been developed to mimic the flight patterns of birds, insects, and bats. However, thanks to the breakthrough of MEMS and artificial intelligence technology, bionic flight vehicles of dragonflies, bees, flies, butterflies, bats and other insects have been developed [4]. They are of the same order of magnitude, with a comparable Reynolds number, and fully in line with the prototype requirements of MAV design. Due to their unique bionic characteristics and flight mode, the flapping-wing aircrafts have great potential in both military and civilian applications. Military applications include enemy reconnaissance, relay communication, electronic interference, and postwar damage assessment. Civilian applications include urban surveillance, road traffic monitoring, agricultural surveys, large-scale patrols, environmental monitoring, disaster monitoring, border patrol and control, and aerial photography [5, 6].

Due to the huge potential of flapping-wing aircrafts, many researches have been carried out. Beetles (Coleoptera) can fold the flexible membrane wing under the sheath wing and can penetrate into the soil and sink into the water, while their hind wings have characteristic, such as large folding rates, which have prompted many researchers to focus on foldable wing. For example, Haas et al. [7] studied the basic principle of folding of beetle rear wings. The folding of the apical region of the hind wing is related to one or several sets of four creases intersecting at a common point. Muhammad et al. [8] used the *Trypoxylus dichotomus* (Coleoptera) as a biomimetic object, dissected the structure of the hind wings, and analyzed the folding and unfolding characteristics. Two prototypes of artificial wings were developed by Muhammad et al. [9]. Jin et al. [10] obtained the external contour and wing parameters of the beetle wing using a scanner and developed a two-dimensional CAD model of the wing. On this basis, a finite element model for aerodynamic simulation was established, and the influence of the interlaced region of the wing vein on the finite element model was analyzed. Nguyen et al. [11] analyzed the fluttering behavior of the beetle and designed a beetle-like flapping-wing aircraft. However, experiments verified that the aircraft did not have enough aerodynamic force to achieve flight. Truong et al. [12] used two simultaneous high-speed cameras to digitize the points marked on the hind wings of the *Trypoxylus dichotomus*, thus achieving a three-dimensional reconstruction of the hind wing motion. The data indicated that the beetle rear wing has more pronounced flexibility and deformation characteristics than other insects. Le et al. [13, 14] performed two-dimensional and three-dimensional CFD (Computational Fluid Dynamics) numerical simulations of beetle hind wing flapping and studied the effects of local corrugation and camber changes on flapping wing aerodynamics. Moreover, they performed a three-dimensional CFD numerical simulation of *Trypoxylus dichotomus*. The synergistic interaction between the hind wing and the sheath wing was found to increase the vertical lift by 6%, thereby supporting the insect's weight. Wang et al. [15] established the physical model of the beetle-folding four-plate wing. The dynamic simulation results show that, with the increase of the wing flapping speed, the instability of the flapping motion during the take-off phase will increase, but it will eventually stabilize, and the overall stabilization time will be shorter.

The above studies demonstrated that current research is mainly focused on the mechanical design and simulation of beetle-like flapping-wing aircrafts and the aerodynamic analysis of forward flight and hovering. However, gliding is another skill that nature has provided to birds and insects, which is the most labor-saving of all flying movements. Jiang [16] conducted a dynamic simulation of the “Flying Wing-Gliding-Flapping-Gliding” motions of birds and found that the flapping-wing aircraft could continuously fly forward in the proposed gliding way, providing good aerodynamic performance. The gliding performance of insects is not superior to that of birds. Among them, the dragonfly has the best characteristics; thus, it is the most studied. Wakeling and Ellington [17] recorded the motion parameters of the dragonfly during free gliding movement using a high-speed camera. The gliding lift-to-drag ratio of the dragonfly was calculated under steady state and was found much greater than that of other insects. The studies of Kesel [18], Vargas [19], and Kwok [20] on dragonfly pleated wings have shown that the pleated airfoil has a higher lift-to-drag ratio than the flat airfoil. Liu et al. [21] studied the intermittent flapping flight performance of dragonfly during climbing and found that the combination of fluttering and gliding can improve the flight performance of bionic aircrafts.

This study is mainly focused on the bionic foldable wings of the beetle. Since the beetle is a large insect, its gliding performance is not clear and little research has been conducted. However, the design of a bionic beetle aircraft with gliding and fluttering functions is of great significance. Such a bionic aircraft, employed with gliding and fluttering functions, can effectively reduce energy consumption and can fly farther and longer. On this basis, in the present study, a four-plate folding wing aircraft that mimics the beetle motion and simulates its gliding process was designed, aiming to improve the flight performance of the aircraft.

## 2. Structural Design of a Bionic Flapping Aircraft with Foldable Beetle Wings

### 2.1. The General Structure of the Foldable-Wing Aircraft

In this study, a bionic flapping aircraft with four-degree-of-freedom beetle foldable wings was designed. As shown in Figure 1, the aircraft consisted of a four-plate folding wing module, a folding wing bracket module, a wing abduction/adduction motion drive module, a folding wing drive module, a pitch drive module, and a tap drive module. In addition, due to its modular design, the mechanism and motion functions of the microflying aircraft have more room for expansion.

### 2.2. Flapping Motion Mechanism

In nature, insects fly through the flapping motion. Based on the anatomy and the motion analysis of *Trypoxylus dichotomus*, the crank-sliding mechanism was used to achieve the flapping motion of the bionic aircraft.

As it can be seen in Figure 1, four-plate folding wing module 1 and folding wing bracket module 2 are fixed, so that module 1 follows module 2 for periodic swinging, in order to complete the flapping motion of the aircraft. When a certain speed is reached, the flapping-wing motor stops, and the aircraft changes to glide mode. In addition, the motor of the pitch drive module is powered by the crank connecting rod. The motion is transmitted to the support plate of the flapping drive module, so that the flapping drive module can rotate relative to the pitching motion module, in order to provide the pitching motion of the aircraft body, thereby changing the gliding angle of the aircraft and adjusting its gliding posture.

### 2.3. Wing Folding Mechanism

Insects and birds close their wings when they are at rest. Beetles fold the hind wings in the wing sheath. In order to mimic the folding action of insect wings, the flexible folding method was employed. Flexible hinges were designed to connect the adjacent flaps of the four-plate folding wings, increasing the reliability during operation and flight.

The folding module can be observed in Figure 2. The wing is folded by a flexible cable. One end of the flexible drive cable of the left folding wing is fixed on a fixing pin (1) on the four-plate folding wing module and sequentially passes through the cable hole on the folding wing attachment, (2) the cable hole of the side member, (3) and the cable hole of the guide column, (4) while the other end of the drive cable is fixed in the groove of the outer wheel (5) of the drive motor. The arrangement and connection of the flexible drive cable on the right folding wing is the same as that on the left folding wing.

The flexible cables of the right and left folding wings are fixed on the same side of the wheel groove, in order to ensure the folding of the wing when the motor-driven flexible cable is tightened. When the folding drive motor rotates clockwise, the flexible cable is tightened, and the four-plate wings are folded. When the folding drive motor rotates counterclockwise, the flexible cable is released, and the four-plate wings unfold by the elastic force of the flexible hinges.

### 2.4. Wing Abduction/Adduction Motion Drive Mechanism

The wing abduction/adduction motion drive module is also driven by a flexible cable. When the abduction/adduction motor rotates counterclockwise, abduction cable I contracts under the driving of the left pin of the reel; at the same time, abduction cable II is released, and abduction cable I pulls the connecting rod, which drives wing abduction. When the connecting rod moves towards the abduction locking position, the wing abduction locking pin is inserted into the abduction locking groove on the lower surface of the connecting rod, thereby achieving wing locking during abduction. When the motor rotates clockwise, adduction cable II contracts under the driving of the left pin of the reel; at the same time, abduction cable I is released, and adduction cable II pulls the connecting rod, which drives wing adduction. When the connecting rod moves towards the adduction locking position, the wing adduction locking pin is inserted into the adduction locking groove on the lower surface of the connecting rod, thereby achieving wing locking during adduction.

The motor of the pitch drive module is powered by the crank connecting rod. The motion is transmitted to the support plate of the flapping drive module, so that the flapping drive module can rotate relative to the pitching motion module, in order to provide the pitching motion of the aircraft body, thereby changing the gliding angle of attack of the aircraft and adjusting its gliding posture.

## 3. Numerical Model of the Bionic Flapping Aircraft

### 3.1. Numerical Simulation Method

The wings of most insects and birds are flexible. In previous studies, the wings have been mostly studied as rigid structures. However, the flexibility of the wings changes the flow field around the wings, and the flow field affects the deformation of the wings, which is a mutual interactive process. In the interactive problem, where both the flow field and the structure are involved, a two-way Fluid-Structure Interaction (FSI) analysis method can obtain more realistic results than a simple flow field analysis.

The fluid analysis software Fluent and the Transient Structural module for finite element numerical calculations of the ANSYS workbench platform were used to establish the two-way Fluid-Structure Interaction numerical model of the foldable wing and simulate its gliding motion. The scheme of two-way fluid-solid coupling calculation can be seen in Figure 3. The fluid calculations were performed in Fluent, and the structural calculations were performed in the Transient Structural module. The System Coupling module was used to contour the fluid-solid coupling surface of the fluid domain and the solid domain and exchange data. When the coupling solution converged, the next calculation was performed.

### 3.2. Calculation Model

In the folding mechanism designed in this paper, the elastic hinge was regarded as a wing vein. When the wing is folded, the elastic hinges store energy, while when the wing is deployed, the elastic hinges release this energy, and the hind wing gradually expands. Since the elastic hinges were attached to the wings, they can be considered as part of the wings. In the folding movement, only the internal force of the wings needs to be considered. The main function of the wing joint mechanism is to drive the abduction and flapping motions. According to the design, the folding movement of the wing is separate from the flapping motion, which helps to improve the control precision of the mechanism. At the same time, it reduces the control difficulty. The core component is the four-plate folding wing module. As it can be observed in Figure 4, the four folding lines intersect at one point, the wing is divided into four parts, and the angles between the each two neighbor lines were *γ*, *δ*, *α*, and *β*, with *δ* + *β* = *γ* + *α* + *π*. Through theoretical research and simulation analysis, it has been found that the folded wing has the maximum folding rate when the angles are *γ* = 63°, *δ* = 94°, *α* = 117°, and *β* = 96° [22]. The designed four-plate wing model is shown in Figure 5. The wing has a half-length of 50 mm, a chord length of 20 mm, and a thickness of 0.2 mm, while the flexible hinge has a length of 4 mm, a width of 2 mm, and a thickness of 0.1 mm.

### 3.3. Computational Model Setup

#### 3.3.1. Parameter Settings of the Fluid Domain

As it can be seen in Figure 6, the designed bionic aircraft is a symmetrical structure. Therefore, in order to save computational resources, the fluid domain was symmetrically developed, and only half of the fluid domain was calculated. The length, width, and height of the fluid domain were selected to be 600, 200, and 400 mm, respectively. The left side was set as the velocity inlet; the right side was set as the pressure outlet; the upper, front, and lower faces were set as static wall faces; and the wing was set as a moving wall face. The flow field in the rear area of the wing is more severe. The far field boundary was set far enough in order to avoid the influence of backflow. Therefore, the wings were placed at a distance of 100 mm from the velocity inlet boundary, which can be used to avoid the influence backflow. Due to the flexible structure of the wing, it will interact with the fluid during flight, which will lead to the deformation of the wing structure. Therefore, a 200 × 100 × 100 mm cuboid mesh refinement area is established near the wing, which is divided by tetrahedral mesh. The advantage of tetrahedral mesh is that it is more suitable for mesh reconstruction and less prone to negative volume. The hexahedral mesh is used in the area far away from the wing, and the mesh deformation is not obvious. The hexahedral mesh has the advantages of less mesh number, good antidistortion performance, short calculation time, and high accuracy. Comprehensive analysis, the tetrahedral mesh and hexahedral mesh are combined to generate the wing's mesh. The total number of meshes is 940000.

Firstly, uncoupled steady calculation is performed until convergence, and the result is taken as the initial value of transient calculation. The order of calculation is to calculate the flow field at first in fluent and then calculate the structure in ANSYS mechanical.

The parameters of the solver were set as follows:

Solver: pressure-based unsteady transient solver;

Turbulence model: RNG K-model, enhanced wall function;

Material properties: air density 1.225 kg*/*m^3^, viscosity 1.7894*e*^−5^ kg/m^−^s;

Boundary conditions: inlet flow rate 1 m*/*s, and the outlet is a pressure outlet;

Dynamic mesh settings: The mesh update method was applied for mesh smoothing and remeshing. And all the surfaces of the wings were set as the fluid-solid coupling surfaces;

Solution method setting: The first-order upwind scheme of SIMPLEC the algorithm was chosen.

#### 3.3.2. Parameter Settings of the Solid Domain

The four-plate folding wing was the structural domain to be solved. The four plates of the wing were connected by four elastic hinges with the same parameters; thus, band constraints were imposed on the wings and each elastic hinge in the Transient Structural module. A fixed constraint was applied on the wing surface, and the gravity acceleration was set vertically downward, and all faces were set as fluid-solid coupling faces. The material parameters of the four plates were defined as *ρ* = 2000 kg/m^3^, *E* = 350 GPa, and *μ* = 0.307, and the parameters of the elastic hinge were defined as *ρ* = 1980 kg/m^3^, and *μ* = 0.3. Based on the elastic modulus of ionic polymer-metal composites (IPMC) in the literature [23], the elastic modulus *E* was set as 1.5 GPa, 2.0 GPa, and 2.5 GPa, respectively. The four-plate folding wings were meshed using a hexahedral mesh, and the number of elements was about 6000.

#### 3.3.3. Fluid-Structure Coupling Settings

In the System Coupling module, the flow field and the surface of the structure are in one-to-one correspondence, so that the fluid solver can exchange data with the structural solver, and vice-versa. In the coupling order, the structural calculation was performed first and the flow field calculation followed.

#### 3.3.4. Lift Coefficient and Drag Coefficient

During gliding, the air flows through the wings, and the wings are subjected to several forces. The force acting on the wing perpendicular to the direction of the incoming flow is called lift force, denoted by *F*_l_, and the force parallel to the direction of the incoming flow is called drag force, denoted by *F*_d_. In order to compare the lift and drag forces under different conditions, the dimensionless lift and drag coefficients are generally calculated. The lift coefficient *C*_l_ and the drag coefficient *C*_d_ are defined as follows [24]:

(1) $$\begin{array}{c} C_{\text{l}}=\frac{F_{\text{l}}}{0.5{pv}^{2}S}\;C_{\text{d}}=\frac{F_{\text{d}}}{0.5{pv}^{2}S}, \end{array}$$

where *ρ* is the density of air, *v* the velocity of air flow, and *S* is the area of the wings.

## 4. Results and Discussion

### 4.1. Effect of Elastic Modulus on the Aerodynamic Performance

The influence of the flexible hinges with different stiffness on the aerodynamic characteristics of the foldable wing was analyzed. The gliding angle of attack was set to 15°, and the elastic modulus *E* was set as 1.5 GPa, 2.0 GPa, and 2.5 GPa.

During gliding, the wing is affected by both aerodynamic forces and its own deformation. In the initial stage, the wing vibrated up and down, then the amplitude of the oscillation became smaller and smaller, and the state of the wing stabilized as the time increased. The change of the lifting resistance in the gliding state is closely related to the deformation and oscillation of the flexible wing and the flexible hinge. Figures 7 and 8 show the change of the lift coefficient and the resistance coefficient of the four-plate folding wing with elastic hinges of different stiffness during the gliding process, respectively. It can be seen that the amplitude of the lift and drag coefficients oscillated with time. When the elastic modulus of the elastic hinge is high, the amplitude of the resistance coefficient is smaller, and thus, the flight state can be more stable. Lift-to-drag ratio is the ratio of the lift coefficient to the drag coefficient during flight. It is an important parameter that indicates the aerodynamic efficiency of the aircraft. In general, the greater the lift-to-drag ratio, the higher the aerodynamic efficiency of the aircraft.  Figure 9 shows the lift-to-drag ratio of the foldable wing with different elastic hinge moduli. It can be seen that due to the small size of the aircraft, the low flight velocity, and the small Reynolds number of the flow field, the elastic modulus of the elastic hinge has little effect on the flow field. The lift-to-drag ratio was between 3.2 and 3.3. Through comprehensive consideration, an elastic modulus of 2.0 GPa was selected for the flexible hinge.

### 4.2. Effect of Attack Angle on the Aerodynamic Performance

The foldable wing designed in this study is a constant-thickness symmetrical airfoil. When the angle of attack is zero and the direction of the inflow is horizontal, the lift force of the foldable wing is close to zero. Therefore, in order to enable the aircraft to generate lift when gliding, the cross-section of the foldable wing needs to have a certain angle with the direction of the incoming flow. The variation of the lift and drag coefficient of a rigid and a flexible foldable wing for attack angles of 2.5°, 5°, 7.5°, 10°, 12.5°, and 15° was analyzed.

In the rigid foldable wing case, the wing does not deform under the aerodynamic forces, and the airflow is stable. Therefore, no fluid-solid coupling problem is involved. When the flow field was stable, the lift and drag coefficients were constant (Figure 10). The lift coefficient and drag coefficient of the rigid wing increased with the increase of the angle of attack. The lift coefficient demonstrated a linear trend. The drag coefficient changed slowly under low attack angles (2.5°-7.5°) and gradually increased as the attack angle increased.

Figures 11 and 12 show the lift and drag coefficient curves of the flexible wing under different angles of attack. It can be seen that the lift and drag coefficients increased with the increase of the angle of attack, and after a period of oscillations, tended to be stable. Thus, the aerodynamic characteristics of flexible wings are different from rigid wings.

The lift-to-drag ratio of the flexible and rigid wings at different attack angles can be seen in Figure 13. When the angle of attack was between 2.5° and 10° (2.5° intervals), the lift-to-drag ratio of the rigid wing increased with the increase of the angle of attack, and the rate of change decreased. When the angle of attack was greater than 10°, the lift-to-drag ratio decreased with the increase of the angle of attack. The trend of the lift-to-drag ratio curve of the flexible wing was the same with that of the rigid wing. The rigid and flexible wings demonstrated the maximum lift-to-drag ratio at 10°. When the angle of attack was 2.5° and 5°, the lift-to-drag ratio of the flexible wing was greater than that of the rigid wing. When the angle of attack was greater than or equal to 10°, the lift-to-drag ratio of the rigid wing was greater than that of the flexible wing, but the difference was small. Thus, it is feasible to design the wings to be flexible. In addition, the angle of attack was found to have little effect on the oscillation stabilization time of the wing, while the lift and drag coefficients tend to be stable after a certain period of time. Taking these two aspects into consideration, the aircraft has a superior aerodynamic performance with a flexible hinge and a gliding angle of attack of 10°.

According to formula (1) and based on the selected structural parameters of the bionic aircraft, the lift was calculated to be approximately 70 mg. It also indirectly indicated that as a heavy insect, the beetle can only fly in a fluttering manner, and its gliding performance is not superior. According to the literature, the Micromechanical Flying Insect (MFI) developed by the University of California at Berkeley is 10-25 mm in size and weighs about 8-43 mg. The Robobee developed by the Harvard Wood Research Group is about 15 mm in size and weighs 60 mg. MEMS technology has been used to achieve miniaturization and weight reduction of these two aircrafts. Therefore, in order to achieve flight modes combined with gliding and fluttering in the bionic aircraft, one solution is to replace the existing mechanical structure with the more advanced and sophisticated MEMS technology and use lighter wing materials. Such an aircraft cannot complete the gliding motion at a gliding speed of 1 m/s (The speed of the beetle's forward flight is roughly 1.5 m/s [14], thus the gliding speed is set to 1 m/s.). The performance of bionic aircrafts can be improved compared to beetles. If an aircraft with higher flying velocity can be designed, and thus, it is possible to achieve gliding. Similar to the Chinese kite, it is difficult to fly under windless conditions. Under the traction produced by the operator, the kite is given a sufficient initial velocity to float in the air. As the height and the wind speed increase, the kite can glide under its own gravity, aerodynamics, and traction in the line. Based on the same principle, if the forward speed of the designed bionic aircraft is improved, the initial speed of the gliding will increase, and thus, sufficient aerodynamic force can be generated to support its gliding. The flight performance of the flexible wings at different inflow speeds under a 10° angle of attack was numerically simulated and analyzed.

Figures 14 and 15 show the lift and drag coefficient curves of the flexible wing under gliding speeds of 1 m/s, 3 m/s, 5 m/s, and 7 m/s. When the gliding speed was 1 m/s, that is, when the Reynolds number was 1333, the lift and drag coefficients oscillated significantly. After 0.5 s, the oscillation of the curve decreased, but its amplitude was still the largest among the four gliding speed levels. When the speed increased to 3 m/s, 5 m/s, and 7 m/s, the lift and drag coefficient curves were different from that at 1 m/s. Before 0.15 s, the curves demonstrated large oscillation, and the intensity of the oscillation was proportional to the gliding speed. The larger the gliding speed, the more severe the oscillation in the early stage of gliding. Then, the curves became quickly stable and approximated a straight line. At different gliding speeds, the lift coefficient was not much different, and the average gliding lift coefficient was around 0.55. The changes in the drag coefficient were more obvious. As the gliding speed increased, the drag coefficient decreased. The lift-to-drag ratio curve is shown in Figure 16. As the gliding speed increased, the lift-to-drag ratio also increased, the aerodynamic efficiency of the aircraft also increased, but the slope of the change gradually decreased. Since the gliding speed directly determines the magnitude of the aircraft aerodynamics, while improving the aerodynamic efficiency, the performance of the aircraft drive is also necessary to be taken into account.

Figure 17 shows the lift of the aircraft at different gliding speeds. It can be seen that as the speed increased, the lift magnitude increased. When the gliding speed was 7 m/s, the lift force of the aircraft was about 0.034 N, which was converted into a weight of about 3.4 g. The class of the aircraft is similar to that of the DelFly Micro developed by the David Research Group at the Delft University of Technology in the Netherlands. The DelFly Micro has a length of 10 cm and a weight of 3.07 g. A micromotor is used to successfully drive the four-bar mechanism [25]. Therefore, if the aircraft designed in this paper can control a weight of about 3 g, then it can also perform the gliding action. The simulation results yielded the minimum lift required to achieve gliding at different speeds. These results can guide the improved design of the structure and weight of the bionic aircraft, achieve flight modes combined with fluttering and gliding, and improve the flight performance of the aircraft.

### 4.3. Flow Field Analysis

Figure 18 present the velocity contours on a span-wise cross-section at different speeds after gliding for 0.5 s. The cross-section is in the middle of the wing tip and the wing root. It can be seen from the velocity contours that the highest velocity was developed at the front edge of the wing. The velocity of the flow on the upper surface of the wing was high, and a high-speed vortex was formed at the leading edge. Such vortices form low-pressure regions. The velocity of the flow at the lower surface of the wing was low, and a high-pressure zone was formed at the leading edge of the lower surface. The velocity contours at different inflow speeds were very similar, and only differences in magnitude were found due to the different speeds.

Figure 19 present the pressure contours on a span-wise cross-section at different speeds after gliding for 0.5 s. As it can be seen, the highest and lowest points of the relative pressure on the wing surface were found at the leading edge of the wing. Due to the difference in speed between the upper and lower surfaces, the pressure under the airfoil was greater than that over the airfoil, which was also lower than the standard atmospheric pressure. The pressure difference between the upper and lower airfoil surface leads to an upward force exerted on the wing, thereby generating lift. The greater the inflow velocity, the greater the pressure difference, and the greater the lift that can be produced, which is consistent with the lift curve characteristics shown in Figure 17.

## 5. Conclusion

1. Based on beetle characteristics, such as the foldable wings and the large folding rate, a bionic foldable flapping wing aircraft was designed. A two-way Fluid-Structure Interaction numerical simulation method was used, and the aerodynamic characteristics of the aircraft in gliding flight were analyzed. The lift and drag coefficients of the foldable wing with different elastic modulus were analyzed. It was found that the elastic modulus of the flexible hinges has little effect on the aerodynamics of the aircraft. Through comprehensive consideration, a material with an elastic modulus of 2.0 GPa was selected for the flexible hinges
2. The gliding performance of rigid and flexible wings under different angles of attack was simulated. The results demonstrated that both the rigid and the flexible wing exhibit the maximum lift-to-drag ratio when the angle of attack is 10°, which provides also a reference for the design of bionic flapping aircrafts
3. Numerical simulations and analysis of the flight performance of the flexible wings at different gliding speeds were carried out. It was found that the magnitude of the lift force increased with the increase of the gliding speed. The lift force was about 0.034 N when the gliding speed was 7 m/s. In order to achieve gliding, it is necessary to improve and simplify the structure of the existing bionic aircraft, use new lightweight materials, and use MEMS technology to decrease the weight and improve the aerodynamics of the aircraft

In the present study, only the gliding state of a single wing was considered, while when insects fly, the two wings are combined in fluttering and gliding modes. Therefore, a future study will incorporate the complete model of the aircraft, simulate the flutter-gliding-flutter flight mode of the bionic aircraft, and analyze the flow field changes during flight and the aerodynamic performance of the aircraft.

## Figures and Tables

**Figure 1:** Main view of the aircraft structural model. 1. Four-plate folding wing module. 2. Folding wing bracket module. 3. Abduction/adduction motion drive module. 4. Folding wing drive module. 5. Pitch drive module. 6. Flapping wing drive module.

**Figure 2:** 3D model diagram of the folding drive module. 1. Fixing pin. 2. Cable hole of the folding attachment. 3. Cable hole of the side member. 4. Cable hole of the guide column. 5. Outer wheel.

**Figure 3:** Scheme of the bidirectional fluid-solid coupling calculation.

**Figure 4:** Theoretical model of the four-plate folding wing.

**Figure 5:** Geometry model of the four-plate folding wing.

**Figure 6:** Gliding state flow field model.

**Figure 7:** Drag coefficient using flexible hinges with different elastic modulus.

**Figure 8:** Lift coefficient using flexible hinges with different elastic modulus.

**Figure 9:** Lift-to-drag ratio versus the elastic modulus of the elastic wing hinges.

**Figure 10:** Lift coefficient and drag coefficient curves for different angles of attack.

**Figure 11:** Lift coefficient curves of the rigid wing under different angles of attack.

**Figure 12:** Drag coefficient curves of the flexible wing under different angles of attack.

**Figure 13:** Lift-to-drag ratio of the rigid and flexible wings for different angles of attack.

**Figure 14:** Lift coefficient of flexible wings at different gliding speeds.

**Figure 15:** Drag coefficient of flexible wings at different gliding speeds.

**Figure 16:** Lift-to-drag ratio of flexible wings at different gliding speeds.

**Figure 17:** Lift of flexible wings at different gliding speeds.

**Figure 18:** Flow field velocity contours (unit: m/s).

**Figure 19:** Flow field pressure contours (unit: Pa).

## Data Availability

The data used to support the findings of this study are available from the corresponding author upon request.

## Notation

*α*, *β*, *γ*, *δ*: The angles between each two neighbor lines
*C*_l_: Lift coefficient
*C*_d_: Drag coefficient
*ρ*: Air density (kg/m^3^)
*V*: The velocity of air flow
*S*: The area of the wing
*L*/*D*: Lift-to-drag ratio.
